The article "Palmitate induces cisternal ER expansion via the activation of XBP-1/CCTα-mediated phospholipid accumulation in RAW 264.7 cells" was published in 2015. Journal: Lipids Health Dis.

# Palmitate induces cisternal ER expansion via the activation of XBP-1/CCTα-mediated phospholipid accumulation in RAW 264.7 cells

**DOI:** 10.1186/s12944-015-0077-3

**Published:** 2015-07-16

**Authors:** Seong Keun Kim, Eunhye Oh, Mihee Yun, Seong-Beom Lee, Gue Tae Chae

**Affiliations:** Institute of Hansen’s Disease, Department of Pathology, College of Medicine, The Catholic University of Korea, 222 Banpo-daero, Seocho-gu, Seoul 137-701 Republic of Korea

**Keywords:** Palmitate, ER expansion, XBP-1, CCTα, Phospholipid accumulation, RAW 264.7 cell

## Abstract

**Background:**

Endoplasmic reticulum (ER) stress induces ER expansion. The expansion of the intracisternal space of the ER was found in macrophages associated with human atherosclerotic lesions. We also previously reported that palmitate induces cisternal ER expansion and necrosis in RAW 264.7 cells. In this study, we report on an investigation of the likely mechanism responsible for this palmitate-induced cisternal ER expansion in a mouse macrophage cell line, RAW 264.7 cells.

**Methods:**

RAW 264.7 cells were pre-treated with the designated inhibitor or siRNA, followed by treatment with palmitate. Changes in the ER structure were examined by transmission electron microscopy. The induction of ER stress was confirmed by an increase in the extent of phosphorylation of PERK, the expression of BiP and CHOP, and the splicing of XBP-1 mRNA. Phospholipid staining was performed with the LipidTOX Red phospholipidosis detection reagent. Related gene expressions were detected by quantitative real time-RT-PCR or RT-PCR.

**Results:**

Palmitate was found to induce ER stress and cisternal ER expansion. In addition, palmitate-induced cisternal ER expansion was attenuated by ER stress inhibitors, such as 4-phenylbutyric acid (4-PBA) and tauroursodeoxycholic acid (TUDCA). The findings also show that palmitate induced-mRNA expression of *CCTα*, which increases phospholipid synthesis, was attenuated by the down-regulation of XBP-1, a part of ER stress. Furthermore, palmitate-induced phospholipid accumulation and cisternal ER expansion were attenuated by the down-regulation of XBP-1 or CCTα.

**Conclusions:**

The findings reported herein indicate that palmitate-induced cisternal ER expansion is dependent on the activation of XBP-1/CCTα-mediated phospholipid accumulation in RAW 264.7 cells.

## Background

Elevated serum free fatty acids (FFAs) in patients with obesity and type 2 diabetes inappropriately accumulate in non-adipose tissue, leading to cellular dysfunction and cell death [1]. Of the various FFAs, palmitate (C16:0) is one of the most abundant saturated fatty acids in plasma [2] and has been reported to be toxic to cardiomyocytes [3] and macrophages [4].

The article "Palmitate induces cisternal ER expansion via the activation of XBP-1/CCTα-mediated phospholipid accumulation in RAW 264.7 cells" was published in 2015. Journal: Lipids Health Dis.

Palmitate has been reported to induce the production of intracellular reactive oxygen species (ROS) generation, which subsequently leads to endoplasmic reticulum (ER) stress and ER expansion in BRIN-BD11 pancreatic β-cells and C2C12 myoblasts [5, 6]. We have also previously reported that palmitate induces cisternal ER expansion in mouse macrophage cell line, RAW 264.7 cells [7]. However, the mechanism of how palmitate induces ER expansion is uncertain in macrophages.

ER stress is one of features shown in lipid-laden macrophages of atherosclerotic plaques [8–10]. ER stress is generally thought to induce ER expansion via unfolded protein response (UPR)-mediated lipid biosynthesis and the subsequent enlargement of the ER, which, in turn, alleviates ER stress [11].

It has been reported that a branch of the UPR induces mRNA splicing which then modifies the X-box binding protein (XBP)-1 transcript, resulting in the expression of the transcription factor, XBP-1(S) [12, 13]. XBP-1(S) is a functionally active transcription factor, whereas the isoform XBP-1(U), encoded by the unspliced mRNA, is devoid of transcriptional activity [14, 15]. In turn, the XBP-1(S) leads an enhancement in the activities of choline cytidylyltransferase (CCT) α and choline phosphotransferase (CPT), thereby increasing the synthesis of phosphatidylcholine (PtdCho), the primary phospholipid of the ER membrane, subsequently leading to ER biogenesis or expansion in NIH-3T3 fibroblasts [12, 13]. Thus, we hypothesized that palmitate-induced cisternal ER expansion may be mediated by XBP-1/CCTα-mediated phospholipid accumulation in macrophages.

The purpose of this study was to investigate the mechanism responsible for the palmitate-induced cisternal ER expansion in RAW 264.7 cells. We initially examined the issue of whether palmitate-induced ER expansion is dependent on ER stress. We also assessed whether palmitate-induced cisternal ER expansion is dependent on the activation of XBP-1/CCTα-mediated phospholipid accumulation.

## Results

### Palmitate induces cisternal ER expansion in RAW 264.7 cells

We previously reported that treatment with palmitate induced necrotic cell death [7]. As shown in Fig. 1a, cells that had been treated with 400 μΜ palmitate mainly showed necrotic characteristics, including a loss of plasma membrane integrity and intracellular vesicle swelling. We also evaluated the apoptotic activity of palmitate by measuring the uptake of APOPercentage dye (red, APOPercentage™ apoptosis assay kit). Staurosporine, a known inducer of apoptosis, was used as a positive control for apoptosis. The palmitate-treated cells showed a similar level of APOPercentage dye uptake compared to control cells, whereas staurosporine-treated cells showed a higher level of APOPercentage dye uptake than control cells (Fig. 1b). Furthermore, the palmitate-treated cells showed a 34.4 % labeling of PI and minimal labeling of annexin V (Fig. 1c).

The article "Palmitate induces cisternal ER expansion via the activation of XBP-1/CCTα-mediated phospholipid accumulation in RAW 264.7 cells" was published in 2015. Journal: Lipids Health Dis.

**Fig. 1:** Palmitate induces necrosis in RAW 264.7 cells. Cells were treated with palmitate at the indicated concentration or 4 μM staurosporine for 24 h. Changes in ER structure were examined by transmission electron microscopy (**a**). The treated cells were stained with the APOPercentage dye (APOPercentage™ kit, Biocolor, Belfast, NIreland) for 1 h (**b**) and, by annexin V-FITC/propidium iodide (PI) and were analyzed by flow cytometry (**c**)

Interestingly, ER expansion was frequently found in cells that survive exposure to palmitate (Figs. 1a and 2). ER expansion was first observed at 4 h after the palmitate treatment and the extent of ER expansion was gradually increased in a dose- and a time-dependent manner in palmitate-treated cells (Fig. 2a and b). In addition, Calnexin, an ER lectin that mediates protein folding on the rough ER [16], was localized on the membrane of cisternal expanded ER (Fig. 2c). These results suggest that palmitate induces the cisternal expansion of rough ER.

**Fig. 2:** Palmitate induces cisternal ER expansion in RAW 264.7 cells. Cells were treated with palmitate at the indicated concentration for 24 h (**a**) and with 400 μM palmitate for the indicated times (**b**). Changes in ER structure were examined by transmission electron microscopy (**a** and **b**). Immunogold staining of calnexin was performed on ultrathin sections of cryoprocessed RAW 264.7 cells (**c**)

### Palmitate-induced cisternal ER expansion is dependent on ER stress in RAW 264.7 cells

We initially investigated the underlying mechanism of palmitate-induced ER expansion in RAW 264.7 cells. As shown in Fig. 3, the ER stress markers such as phosphorylated PERK, BiP, CHOP, and spliced XBP-1 mRNA were increased after treatment with palmitate in a dose- or time- dependent manner. In addition, we examined the effect of ER stress inhibitors, 4-PBA and TUDCA, on the palmitate-induced cisternal ER expansion. It has been reported that 4-PBA and TUDCA are chemical chaperones and reduce ER stress by improving ER folding capacity and by blocking a calcium-mediated apoptotic pathway, respectively [17, 18]. Pre-treatment with the above ER stress inhibitors resulted in the attenuation of palmitate-induced ER stress (Fig. 4a and b) and cisternal ER expansion (Fig. 4c). These results suggest that palmitate-induced cisternal ER expansion is dependent on ER stress in RAW 264.7 cells.

The article "Palmitate induces cisternal ER expansion via the activation of XBP-1/CCTα-mediated phospholipid accumulation in RAW 264.7 cells" was published in 2015. Journal: Lipids Health Dis.

**Fig. 3:** Palmitate induces ER stress in RAW 264.7 cells. Cells were treated with palmitate at the indicated concentration for 24 h (**a** and **b**) and with 400 μM palmitate for the indicated times (**c** and **d**). The phosphorylation of PERK, and the expression of BiP and CHOP were determined by western blot analysis (**a** and **c**). Total RNA was extracted and reverse transcribed to cDNA. Full-length and spliced *XBP-1* cDNAs were amplified by PCR with mouse *XBP-1* primers. *Gapdh* cDNA was included as an internal loading control (**b** and **d**)

**Fig. 4:** Palmitate-induced cisternal ER expansion is dependent on ER stress in RAW 264.7 cells. Cells were pre-treated with or without 4 mM 4-PBA or 40 μM TUDCA for 1 h and followed by treatment with 400 μM palmitate for 24 h. The phosphorylation of PERK, and the expression of BiP and CHOP were determined by western blot analysis (**a**). Total RNA was extracted and reverse transcribed to cDNA. Full-length and spliced *XBP-1* cDNAs were amplified by PCR with mouse *XBP-1* primers. *Gapdh* cDNA was included as an internal loading control (**b**). Changes in ER structure were examined by transmission electron microscopy (**c**)

### Palmitate induces phospholipid accumulation in RAW 264.7 cells

It has been reported that the increased phospholipid of the ER membrane leads ER expansion in mouse C2C12 myoblasts [6]. We thus examined the effect of palmitate on phospholipid accumulation in RAW 264.7 cells. As shown in Fig. 5, phospholipid (red fluorescence) was accumulated and distributed mainly around ER labeled with anti-calnexin antibody (green fluorescence) in palmitate-treated RAW 264.7 cells.

**Fig. 5:** Palmitate induces phospholipid accumulation in RAW 264.7 cells. Cells were treated with 400 μM palmitate or 10 μg/ml tunicamycin for 24 h and then subjected to immunofluorescence using calnexin antibody and LipidTOX Red dye to examine phospholipid accumulation in ER. Green fluorescence indicates calnexin or ER membrane, red fluorescence indicates phospholipids and yellow fluorescence indicates co-localization of phospholipids with ER membrane

### Palmitate-induced cisternal ER expansion is dependent on the activation of XBP-1/ CCTα-mediated phospholipid accumulation in RAW 264.7 cells

XBP-1(S), a transcription factor translated by splicing *XBP-1* mRNA, has been reported to induce the activation of choline cytidylyltransferase (CCT) α and choline phosphotransferase (CPT), thereby increasing the synthesis of phospholipid in the ER membrane, subsequently leading to ER expansion in NIH-3T3 fibroblasts [12, 13]. Thus, we hypothesized that palmitate-induced cisternal ER expansion may be mediated by XBP-1/ CCTα-mediated phospholipid accumulation. We initially examined the effect of XBP-1 on CCTα-mediated phospholipid accumulation in RAW 264.7 cells. As shown in Fig. 6, treatment with palmitate increased the expression of *CCTα* at mRNA and protein levels and the down-regulation of XBP-1 by *XBP-1* siRNA transfection inhibited palmitate-induced *CCTα* mRNA expression. In addition, the down-regulation of XBP-1 or CCTα attenuated palmitate-induced phospholipid accumulation (Fig. 7) and cisternal ER expansion (Fig. 8). These results suggest that palmitate induces cisternal ER expansion via the activation of XBP-1/CCTα-mediated phospholipid accumulation in RAW 264.7 cells.

The article "Palmitate induces cisternal ER expansion via the activation of XBP-1/CCTα-mediated phospholipid accumulation in RAW 264.7 cells" was published in 2015. Journal: Lipids Health Dis.

**Fig. 6:** Palmitate-induced *CCTα* expression is dependent on XBP-1 in RAW 264.7 cells. Cells were transfected with control or *XBP-1* siRNA. After 48 h transfection, the transfected cells were treated with 400 μM palmitate for 24 h. CCTα expression at the mRNA level was determined by quantitative real time RT-PCR (**a**) and at the protein level by western blot analysis (**b**). Similar results were observed in three independent experiments. *P < 0.01 versus non-treated control cells

**Fig. 7:** Palmitate-induced phospholipid accumulation is inhibited by the down-regulation of XBP-1 or CCTα in RAW 264.7 cells. Cells were transfected with control, *XBP-1* or *CCT*α siRNAs. After 48 h transfection, the effect of *XBP-1* or *CCTα* siRNA transfection was confirmed by western blot analysis (**a**). The transfected cells were treated with 400 μM palmitate for 24 h and then subjected to immunofluorescence using calnexin antibody and LipidTOX Red dye to examine phospholipid accumulation in ER. Green fluorescence indicates calnexin or ER membrane, red fluorescence indicates phospholipids and yellow fluorescence indicates co-localization of phospholipids with ER membrane (**b**)

**Fig. 8:** Palmitate-induced cisternal ER expansion is attenuated by the down-regulation of XBP-1 or CCTα in RAW 264.7 cells. Cells were transfected with control, *XBP-1* or *CCTα* siRNAs. After 48 h transfection, the transfected cells were treated with 400 μM palmitate for 24 h. Changes in ER structure were examined by transmission electron microscopy

### Tunicamycin does not induce cisternal ER expansion in RAW 264.7 cells

We also examined the issue of whether ER stress is sufficient to induce cisternal ER expansion in RAW 264.7 cells. We treated cells with tunicamycin, a well-known ER stressor. The ER stress markers such as phosphorylated PERK, BiP, CHOP, and spliced *XBP-1* mRNA were all increased in the tunicamycin-treated cells (Fig. 9a and b).

**Fig. 9:** Tunicamycin does not induces cisternal ER expansion in RAW 264.7 cells. Cells were treated with 10 μg/ml tunicamycin for 24 h. The phosphorylation of PERK, and the expression of BiP and CHOP were determined by western blot analysis (**a**). Total RNA was extracted and reverse transcribed to cDNA. Full-length and spliced *XBP-1* cDNAs were amplified by PCR with mouse *XBP-1* primers. *Gapdh* cDNA was included as an internal loading control (**b**). Changes in the ER structure were examined by transmission electron microscopy (**c**)

Although the tunicamycin treatment induced dilation of the ER (Fig. 9c), it induced less phospholipid accumulation than the palmitate treatment (Fig. 5) and no cisternal ER expansion (Fig. 9c). These results suggest that the tunicamycin-induced ER stress is not sufficient to cause cisternal ER expansion, indicating the important role of palmitate-induced phospholipid accumulation in cisternal ER expansion.

The article "Palmitate induces cisternal ER expansion via the activation of XBP-1/CCTα-mediated phospholipid accumulation in RAW 264.7 cells" was published in 2015. Journal: Lipids Health Dis.

### Palmitate-induced cell death is not rescued by the down-regulation of XBP-1 or CCTα in RAW 264.7 cells

It has been reported that ER stress leads ER expansion, which, in turn, alleviates ER stress [11]. However, if ER expansion is more extended, then ER structure and integrity are disrupted, which subsequently may lead to cell dysfunction or death. We thus examined the effect of inhibition of ER expansion on palmitate-induced cell death in RAW 264.7 cells. Pre-treatment with the ER stress inhibitors, 4-PBA or TUDCA, led to an increase in cell viability in palmitate-treated RAW 264.7 cells (Fig. 10a). However, the down-regulation of XBP-1 by *XBP-1* siRNA transfection aggravated cell death rather than protection from palmitate-induced cell death, while no effect was found in the case of CCTα down-regulation (Fig. 10b). Although the ER stress is responsible for palmitate-induced cell death, these results suggest that ER expansion is not a prerequisite for induction of cell death in palmitate-treated cells (Fig. 11).

**Fig. 10:** Palmitate-induced cell death is not rescued by the down-regulation of XBP-1 or CCTα in RAW 264.7 cells. Cells were pre-treated with or without 4 mM 4-PBA or 40 μM TUDCA for 1 h and followed by treatment with 400 μM palmitate for 24 h (**a**). Cells were transfected with control, *XBP-1* or *CCTα* siRNAs. After 48 h transfection, the transfected cells were treated with 400 μM palmitate for 24 h (**b**). Cell viability was assessed by an MTT assay. *P < 0.01 versus control cells

**Fig. 11:** A schematic diagram of the signaling pathway involved in the palmitate-induced ER stress-mediated ER expansion in RAW 264.7 cells

## Discussion

Plasma FFA levels are increased from basal levels, in the range of 200–400 μΜ up to 800–1500 μΜ in individuals with obesity and type 2 diabetes [19]. The concentration of 400 μΜ, at which palmitate significantly induced cisternal ER expansion in RAW 264.7 cells, would be pathologically relevant in patients with obesity and type 2 diabetes, since the proportion of palmitate in FFAs is about 25 % [2] and plasma FFAs levels increase to 800–1500 μΜ in patients with obesity and type 2 diabetes [19].

The article "Palmitate induces cisternal ER expansion via the activation of XBP-1/CCTα-mediated phospholipid accumulation in RAW 264.7 cells" was published in 2015. Journal: Lipids Health Dis.

In this study, we dissolved palmitate in NaOH/Et-OH rather than conjugating palmitate with BSA and added palmitate-dissolved in NaOH/Et-OH directly to the culture media to reduce the effect of endotoxins, although the proportion of palmitate that is bound to serum albumin or left in an unbound state is unclear when palmitate is directly added to culture media. It has been reported that the problem of endotoxin contamination exists even after using a low-endotoxin preparation of BSA while preparing palmitate/BSA complexes [20]. We also detected endotoxin contamination in palmitate-bound to BSA using the ToxinSensor™ Endotoxin Detection System (GenScript, Piscataway, NJ, USA) (data not shown). Thus, Schwartz et al. [20] recommended a new method for preparing FFA, which we used in this study.

The ER is a continuous membrane organelle that consists of a nuclear envelope and a peripheral network of tubules and sheets, which make up the smooth and rough ER, respectively [21]. It also serves as a principal site for protein synthesis and folding, protein glycosylation, calcium storage and signaling, sterol biosynthesis, and drug metabolism. Thus, the ER is sensitive to alterations in calcium homeostasis and the accumulation of misfolded proteins. The depletion of Ca^2+^, the inhibition of glycosylation, exposure to chemical toxins or reactive oxygen species, and/or the accumulation of misfolded proteins in the ER lead to ER stress and sustained ER stress eventually results in cell death [22]. To overcome such ER stress, the ER responds by triggering UPR, the ER-overload response (EOR), and ER-associated degradation (ERAD) [22].

In a branch of the UPR, the ER transmembrane kinase/endonuclease IRE1α and β initiate a novel UPR-mediated mRNA splicing mechanism that modifies XBP-1 transcripts to encode a potent basic leucine zipper transcription factor, XBP-1(S). XBP-1(S) plays an important role in phospholipid synthesis in the ER membrane, especially PtdCho, by activating the CCTα and CPT enzymes. This phospholipid allows ER biogenesis and expansion under conditions of ER stress in NIH-3T3 fibroblasts [12, 13]. ER expansion through the UPR-mediated activation of lipid biosynthesis has been reported to alleviate stress. Schuck et al. [11] reported that treatment with DTT, an inhibitor of disulfide bond formation, causes a massive expansion of the ER through the activation of UPR signaling and the resulting ER expansion, in turn, alleviates stress in *Saccharomyces cerevisiae*. In that report, the authors suggested that the UPR maintains ER homeostasis by providing new ER-folding machinery and by providing additional ER surface area and luminal space. Consistent with this result, our results also show that the inhibition of ER expansion by the down-regulation of XBP-1 by *XBP-1* siRNA transfection aggravated cell death rather than conferred protection from palmitate-induced cell death (Fig. 10b) and that ER expansion was frequently found in cells that survive exposure to palmitate (Figs. 1a and 2), suggesting that ER expansion is induced to reduce ER stress and subsequent cell death in palmitate-treated cells (Fig. 11). Interestingly, the expansion of the intracisternal space of ER was reported in macrophages residing in human atherosclerotic lesions [23]. In atherosclerotic lesions, macrophages are recruited to the lesions and engulf excess lipids such as saturated fatty acids or free cholesterol, and eventually undergo ER stress. However, if the ER stress is extended further, it then induces macrophage death via UPR signaling, thereby resulting in necrotic core formation and plaque destabilization [24].

The article "Palmitate induces cisternal ER expansion via the activation of XBP-1/CCTα-mediated phospholipid accumulation in RAW 264.7 cells" was published in 2015. Journal: Lipids Health Dis.

In addition, ER stress is also associated with insulin resistance, which is a major characteristic of metabolic diseases such as obesity and type 2 diabetes. It has been reported that ER stress inhibits insulin receptor signaling via the promotion of the c-Jun N-terminal kinase (JNK)-dependent serine phosphorylation of insulin receptor substrate (IRS)-1, subsequently leading to insulin resistance in mouse models of obesity [25]. Peng et al. [6] also reported that treatment with palmitate induced ER stress and reduced insulin-stimulated Akt phosphorylation. In that report, the authors showed that pre-treatment with 4-PBA, an inhibitor of ER stress, efficiently reversed the suppression of Akt phosphorylation by palmitate treatment in a mouse skeletal muscle cell line, C2C12 cells, suggesting that ER stress is a key event linking high plasma FFA concentrations and insulin resistance in skeletal muscle.

The findings reported herein clearly show that treatment with 400 μΜ palmitate induced cisternal ER expansion and ER stress in RAW 264.7 cells (Figs. 2 and 3). Diakoginnaki et al. [5], also reported that treatment with 250 μΜ palmitate induced ER stress and cisternal ER expansion in BRIN-BD11 pancreatic β-cells. In addition, our results indicate that the palmitate-induced ER stress-mediated activation of XBP-1/CCTα/phospholipid accumulation is also involved in cisternal ER expansion (Figs. 7 and 8). However, tunicamycin-induced ER stress is not sufficient to cause cisternal ER expansion, although the tunicamycin treatment induced the splicing of XBP-1 mRNA and ER dilation (Fig. 9). In addition, our results showed that the tunicamycin treatment resulted in a lower accumulation of phospholipid compared to the palmitate treatment (Fig. 5), suggesting that direct palmitate-induced phospholipid accumulation is required for cisternal ER expansion, in addition to the activation of XBP-1/CCTα/phospholipid accumulation.

The article "Palmitate induces cisternal ER expansion via the activation of XBP-1/CCTα-mediated phospholipid accumulation in RAW 264.7 cells" was published in 2015. Journal: Lipids Health Dis.

It has been reported that palmitate induces not only ER stress but also the direct disruption of ER structure. Borradaile et al. [26], reported that treatment with 500 μΜ palmitate induced the generation of intracellular reactive oxygen species (ROS), which subsequently leads to ER stress in Chinese hamster ovary cells and H9c2 cardiomyoblasts. The authors also showed that palmitate was directly incorporated into saturated phospholipids and triglycerides in the ER membrane, resulting in a dramatic dilation in the ER and subsequently cell death in Chinese hamster ovary cells. In that report, the authors suggested that the deleterious effect of palmitate on the ER is twofold: 1) palmitate-induced ROS generation/ER stress/cell death; 2) the incorporation of palmitate into the ER membrane/dramatic changes in ER structure and integrity. It has also been reported that the incorporation of palmitate into phospholipid, such as PtdCho, induces detrimental stiffening of the ER membrane, loss of function, and activates ER stress signaling in rat hepatoma cell line, H4IIEC3 cells [27, 28].

## Conclusions

The findings reported herein indicate that palmitate induces cisternal ER expansion via the activation of XBP-1/CCTα-mediated phospholipid accumulation in RAW 264.7 cells. These findings point to a new mechanism to explain the link between elevated levels of serum FFAs and ER expansion in macrophages.

## Materials and methods

### Reagents and antibodies

Palmitate, 4-phenylbutyric acid (4-PBA), tauroursodeoxycholic acid (TUDCA), and tunicamycin were obtained from Sigma Aldrich Co. Ltd. (St. Louis, MO, USA). 4-PBA, TUDCA and tunicamycin were dissolved in DMSO. The final vehicle concentration was adjusted to 0.1 % (v/v) and the control medium contained the same quantity of vehicle. LipidTOX was obtained from Invitrogen (Carlsbad, CA, USA). Antibodies against phospho-PERK, PERK, BiP and the Alexa Fluor® 488-conjugated secondary antibody were obtained from Cell Signaling Technology (Beverly, MA, USA). Antibodies against CHOP and calnexin were obtained from Abcam (Cambridge, MA, USA). Antibodies against GAPDH and horseradish peroxidase-conjugated secondary antibodies were obtained from Santa Cruz Biotechnology (Santa Cruz, CA, USA). 1.4 nm gold particles conjugated secondary antibody and HQ silver enhancement kit were obtained from Nanoprobes (Stony Brook, NY, USA).

The article "Palmitate induces cisternal ER expansion via the activation of XBP-1/CCTα-mediated phospholipid accumulation in RAW 264.7 cells" was published in 2015. Journal: Lipids Health Dis.

### Cell culture

The RAW 264.7 murine macrophage cell line was acquired from ATCC (Manassas, VA, USA) and grown as described previously [29].

### Palmitate preparation

Palmitate was prepared as described previously [20]. The problem of endotoxin contamination still existed even after using a low-endotoxin preparation of bovine serum albumin (BSA) while preparing palmitate/BSA complexes. Endotoxin was detected in palmitate-bound to BSA using the ToxinSensor™ Endotoxin Detection System (GenScript, Piscataway, NJ, USA). To reduce endotoxin contamination, the palmitate was dissolved to a final concentration of 40 mM in a solvent composed of 0.1 N NaOH/70 % ethanol and added directly to the cell culture media, where it formed a complex with the bovine serum albumin contained by the 10 % fetal bovine serum. The control medium contained the same quantity of the solvent. i.e., 0.1 N NaOH/70 % ethanol.

### Transmission electron microscopy

Cells were fixed with 2.5 % glutaraldehyde for 2 h, post fixed by treatment with 1 % osmium tetroxide, dehydrated in ethanol, and embedded in Epon 812 (Polyscience, Warrington, PA, USA). Ultrathin ections were contrasted with uranyl acetate and lead citrate. The Sections were examined by transmission electron microscopy (JEOL, Arishima, Japan).

### Immunogold electron microscopy

The pre-embedding immunogold-silver technique was performed to detect the calnexin protein. The sections (50 μm thick) were blocked with a PSG solution [0.05 % saponin/0.2 % gelatin/0.01 M phosphate-buffered saline (PBS)] containing 1 % bovine serum albumin and then incubated with a calnexin antibody overnight at 4 °C. The sections were then incubated with a secondary antibody conjugated with 1.4 nm gold particles for 2 h, and silver enhancement was performed with the HQ silver enhancement kit for 3 min. The sections were examined by transmission electron microscopy (JEOL, Arishima, Japan).

### APOPercentage apoptosis assay

Apoptosis was detected using an APOPercentage™ kit (Biocolor, Belfast, NIreland). Phosphatidylserine at the outside surface of the cell membrane allows the unidirectional transport of the APOPercentage dye to the interior of the cell, where it is retained and accumulates as a red-dye in apoptotic cells. The treated cells in 24- or 96-well culture plates were stained with the APOPercentage dye for 1 h. The medium was then removed and cells were washed twice with PBS. Three representative areas from each well were photographed. The levels of APOPercentage dye uptake were quantified by the colorimetric method according to the manufacturer’s instructions.

The article "Palmitate induces cisternal ER expansion via the activation of XBP-1/CCTα-mediated phospholipid accumulation in RAW 264.7 cells" was published in 2015. Journal: Lipids Health Dis.

### Annexin V-PI staining

To investigate the mechanism associated with the death of palmitate-treated cells, the cells were double stained with annexin V/propidium iodide (PI), using Annexin V-FITC Apoptosis Detection Kit (BD Pharmingen, San Diego, CA, USA) and analyzed by flow cytometry.

### Western blotting analysis

At designated times, the treated cells were removed from the incubator and placed on ice. The cells were then washed 3 times with ice-cold PBS. The cells were then lysed for 30 min with RIPA lysis buffer [50 mM Tris–HCl (pH 7.4), 1 % Triton X-100, 150 mM NaCl, 0.1 % SDS, 0.5 % sodium deoxycholate, 100 mM phenylmethylsulfonyl fluoride, 1 μg/ml of leupeptin, 1 mM Na3VO4, and 1× Complete™ Protease Inhibitor Cocktail (Santa Cruz Biotechnology, Santa Cruz, CA, USA)]. Equal amounts of protein were loaded onto 10 - 15 % SDS-PAGE gels, electrophoresed, and transferred onto PVDF membranes (Millipore, Bedford, MA, USA). The membranes were blocked in Tris-Buffered Saline with 0.05 % Tween 20 (TBST) supplemented with 5 % powdered milk or 5 % BSA, and then incubated with primary antibodies against the designated proteins. The blots were then washed with TBST and incubated with a horseradish peroxidase-conjugated secondary antibody in TBST plus a 5 % solution of powdered milk. The bound antibodies were detected with Super Signal Ultra chemiluminescence reagents (Pierce Biotechnology, Inc., Rockford, IL, USA).

### Inhibitor treatment

Cells were plated on 6-well plates. After 24 h, the cells were pre-treated with the designated inhibitors for 1 h, followed by treatment with palmitate at the indicated concentrations. After incubation for the designated times, the cells were harvested for the next experiment. The concentrations of inhibitors used were as follows: 4-PBA, 4 mM and TUDCA, 40 μM. None of the inhibitors used had a significant effect on the viability of RAW 264.7 cells.

### siRNA transfection

For silencing *XBP-1* and *CCTα*, *XBP-1* and *CCTα*-directed siRNA pool (ON-TARGET plus SMARTpool reagent) and control siRNA were purchased from Dharmacon (Lafayette, CO, USA). Cells were transfected with *XBP-1*, *CCTα*, or control siRNA by electroporation under conditions of a voltage of 1350 and 35 ms using a pipette type electroporator (MicroPorator-Mini, Disital Bio Technology, Suwon, Kyounggi-do, Korea) according to the manufacturer’s instructions. The efficiency of *XBP-1* or *CCTα* siRNA transfection was confirmed by western blot analysis at 48 h after transfection.

The article "Palmitate induces cisternal ER expansion via the activation of XBP-1/CCTα-mediated phospholipid accumulation in RAW 264.7 cells" was published in 2015. Journal: Lipids Health Dis.

### Phospholipid staining and Immunostaining

For phospholipid staining, the cells were treated with 400 μM palmitate containing 1X LipidTOX Red phospholipidosis detection reagent. For Immunostaining with an anti-calnexin antibody, the cells were fixed in 4 % paraformaldehyde in PBS. The fixed cells were rinsed with PBS and incubated in blocking solution (5 % goat serum, and 0.001 % Tween-20 in TBS) for 20 min. The cells were then incubated overnight with an anti-calnexin antibody in an incubation solution (5 % goat serum, and 0.1 % Tween-20 in TBS) at 4 °C. After washing with PBS, the cells were incubated with the corresponding Alexa Fluor® 488-conjugated secondary antibody at room temperature for 2 h. Nuclei were counterstained for 15 min with 10 μM Hoechst 33342 (Sigma-Aldrich Co. Ltd). The negative control was processed without the presence of the primary antibody. Immunofluorescence was visualized by inverted fluorescence microscopy (IX71/IX51, Olympus Corporation Corporation, Tokyo, Japan).

### RT-PCR

Total RNA was extracted using a High Pure RNA isolation kit (Roche Diagnostics, Mannheim, Germany) and converted to cDNA using an Advantage RT-for-PCR kit (Clontech, Hampshire, UK), according to the manufacturer’s instructions. The cDNA was then amplified by PCR using the forward primer *XBP1s* (5’-ACC TGA GCC CGG AGG AGA AA-3’) and reverse primer *XBP1a* (5’-GTC CAG AAT GCC CAA AAG GA-3’). GAPDH RNA was amplified using the forward primer *GAPDHs* (5’-GCC TTC CGT GTT CCT ACC-3’) and the reverse primer *GAPDHa* (5’-CCT GCT TCA CCA CCT TCT T-3’). PCR products were separated on a 2.5 % agarose gel.

### Quantitative real time-RT-PCR

The expression of *CCTα* mRNA was determined by quantitative real time-RT-PCR. Briefly, total RNA was extracted using a High Pure RNA isolation kit (Roche Diagnostics, Mannheim, Germany) and converted to cDNA using an Advantage RT-for-PCR kit (Clontech, Hampshire, UK), according to the manufacturer’s instructions. To quantify *CCTα* mRNA, quantitative real time RT-PCR was performed with a iQTM SYBR® Superrmix kit (BIO-RAD Laboratories, Hercules, CA) in a Peltier Thermal Cycler-200 system (MJ Research, Berlin, Germany). Real time PCR was performed in triplicate at 95 °C for 3 min followed by 35 cycles of amplification (94 °C for 30 s, 58 °C for 30 s, and 72 °C for 30 s). The relative amounts of mRNA for *CCTα* was determined by subtracting the cycle threshold (Ct) values for these genes from the Ct values for *Gapdh*. The following primers for *CCT*α and *Gapdh* were used: For *CCTα*, forward primer (5’- GAT GAG CTA ACG CAC AAC TTC AA -3’) and reverse primer (5’- GTG CTG CAC GGC GTC ATA -3’). For *Gapdh*, forward primer (5’-GGG AAG CTC ACT GGC ATG G-3’) and reverse primer (5’-CTT CTT GAT GTC ATC ATA CTT GGC AG-3’).

The article "Palmitate induces cisternal ER expansion via the activation of XBP-1/CCTα-mediated phospholipid accumulation in RAW 264.7 cells" was published in 2015. Journal: Lipids Health Dis.

### Cell viability assay

Cell viability was evaluated by an MTT [3-(4,5-dimethylthiazol-2-yl)-2,5-diphenyltetrazolium bromide] reduction assay in 96-well plates. At designated times, 10 μL of 50 mg/mL MTT solution was added to each well. After incubation in a 5 % CO_2_ incubator for 2 h at 37 °C, the media was removed and 100 μL of acid isopropyl alcohol was added to each well. After 10 min incubation, 100 μL of distilled water was added to each well and the optical density of each well was then measured at 570 nm with a spectrometer (μ-Quant, Bio-tech instrument, Inc., Winooski, VT).

### Statistical analysis

All results are expressed as the means ± S.D. of data from at least three separate experiments. Statistical significance was determined via the Student’s *t*-test for two points. *p* < 0.01 was considered to be statistically significant.

## Abbreviations

FFA: Free fatty acids
CCTα: Choline cytidylyltransferase α
CPT: Choline phosphotransferase
XBP-1: X-box binding protein-1
4-PBA: 4-phenylbutyric acid
TUDCA: Tauroursodeoxycholic acid
PtdCho: Phosphatidylcholine
ROS: Reactive oxygen species
ER: Endoplasmic reticulum
UPR: Unfolded protein response
PERK: Protein kinase RNA-like endoplasmic reticulum kinase
CHOP: CCAAT/-enhancer-binding protein homologous protein
PI: Propidium iodide
MTT: 3-(4,5-dimethylthiazol-2-yl)-2,5-diphenyltetrazolium bromide
